# Influence of Pretreatment System on Inorganic Suspended Solids for Influent in Wastewater Treatment Plant

**DOI:** 10.1155/2022/2768883

**Published:** 2022-09-28

**Authors:** Li He, Yong Zhang, Dan Song, Zhongwen Ou, Zhigang Xie, Subo Yang, Wei Guan, Cunlan Dong, Yifu Zhang

**Affiliations:** ^1^Zunyi Normal University, Resource and Environment College, Zunyi 563006, China; ^2^Chongqing Research Academy of Environmental Sciences, Chongqing 401147, China; ^3^Army Logistics University of PLA, Chongqing 401311, China; ^4^Chongqing University of Arts and Sciences, Chongqing Key Laboratory of Environmental Materials & Remediation Technologies, Chongqing 402160, China; ^5^Chongqing Gangli Limited Corporation, Chongqing 400042, China

## Abstract

In order to investigate the cause of accumulation of the inorganic suspended solid (ISS) in biochemical tank for wastewater treatment plant (WWTP) in recent years, the influent quality of one WWTP in Chongqing was monitored in one year, and the removal efficiency of ISS during the pretreatment process was studied. Results showed that the low removal efficiency of ISS (<7%) was ascribed to the weak removal efficiency of sand in the grit chamber. The primary sedimentation tank showed a good removal efficiency of ISS up to 69% and also had a good removal efficiency of COD up to 70%. The annual variation rule of MLVSS/MLSS for mixed liquor varied in contrast to the influent quality, ranging from 0.24 to 0.57, much lower than the normal value of 0.7. In order to maintain the normal function of activated sludge, it is necessary to retain the primary sedimentation tank to remove ISS.

## 1. Introduction

The pretreatment system of municipal wastewater treatment plant includes grille sand, grit chamber, and primary sedimentation tank, among which the main grit chamber and primary sedimentation tank could remove pollutants, and the treated wastewater directly entered into the biochemical tank. Some research was focused on the influences of influent and flow on the removal efficiency of phosphorus and nitrogen in the biochemical treatment system, obtaining much precious operation regulation experience [1–3]. However, less attention had been paid to inorganic suspended solids in influent. In recent years, a large number of inorganic solids were deposited at the bottom of structures in oxidation ditch and other sewage treatment systems, resulting in reducing the hydraulic retention time of wastewater and the effective volume of reactor, which seriously affected the performance of wastewater treatment [4, 5]. Meanwhile, a large number of studies had shown that MLVSS/MLSS of activated sludge was significantly affected by inorganic solids of influent, and the MLVSS/MLSS of activated sludge in many wastewater treatment plants was as low as 0.3-0.5, which was below the normal level of 0.7 [6–10]. The results indicated that there were still a large number of inorganic suspended solids flowing into the biochemical treatment system after the pretreatment system, reducing the activity of activated sludge. Therefore, the influent quality of one WWTP in Chongqing was monitored in one year, and the removal efficiency of ISS during the pretreatment process was studied. Meanwhile, the influences of the pretreatment system of grit chamber and primary sedimentation tank on the treatment of inorganic suspended solids in sewage were analyzed, providing technical support for solving the problem of the decrease of the organic component ratio of activated sludge.

## 2. Materials and Methods

### 2.1. Sampling Points of the Wastewater Treatment Plant

The wastewater treatment plant was located in the main urban area of Chongqing, and the combined sewerage system was used for sewage collection. The service area of the WWTP was 125 km^2^ with a processing capacity of 60,000 t/d in dry season and 100,000 t/d in rainy season. The pretreatment system for sewage treatment was composed of rotational flow sedimentation tank, horizontal sedimentation tank, and the inverted A^2^O process of biochemical treatment system. And the process flow is shown in Figure 1. Besides, 27 samples were conducted from May 2020 to June 2021, and the sampling points are shown in Figure 1. During the sampling process, a professional bottom inlet water quality sampler was used to take water samples, so as to ensure the representativeness of samples.

### 2.2. Index Analysis

The concentrations of SS, TP, MLSS, TN, and TP were measured by Water and Wastewater Monitoring Methods (4th edition). SS was calcined in muffle furnace at 600°C temperature for 1 h and calcined to constant weight, so the remaining residue was ISS. The particle size distribution in the test sample was analyzed by BT-9300HT laser particle size measurement system (Dandong Better Technology Co., LTD., China), with the measurement range of 0.1~1000 *μ*m.

## 3. Results and Discussion

### 3.1. Removal Performance of Pretreatment System

The mean values of water quality parameters of 27 samples are shown in Table 1, and the removal efficiencies of each pollutant using the pretreatment system are shown in Table 2.

According to the classification of typical domestic sewage by Metcalfe and Eddy company. The concentration of SS and ISS for this sewage factory was higher than the domestic sewage with high intensity. The concentration of SS was reduced to the moderate strength, and the concentration of ISS was still higher than high strength after primary sedimentation treatment. The concentration of COD for influent did not meet the higher strength, while the concentration of COD was lower than the low strength after wastewater treatment.

As shown in Table 1, after the treatment of grit chamber, the average concentration of COD of wastewater was decreased from 635 to 620 mg/L, the average concentration of SS was decreased from 1123 to 1048 m/L, the average concentration of ISS was decreased from 809 to 769 mg/L, and the concentrations of TN and TP were changed little. According to the treatment efficiency in Table 2, it was found that the removal efficiency of each pollutant was less than 7%, indicating that the removal efficiency of pollutants in the grit chamber was weak. In general, the grit chamber had a good removal efficiency of suspended solids with particle size larger than 200 *μ*m. As the particle size of SS for influent in the grit chamber was about 60.93 *μ*m and far less than 200 *μ*m, the removal efficiencies of SS and ISS were very lower.

The average removal efficiencies of COD, SS, ISS, TN, and TP were 55.32%, 69.71%, 69.86%, 29.82%, and 44.83%, respectively. The removal efficiencies of SS and COD in ordinary advection sedimentation tank were about 50% and 30%, and the removal efficiency of pollution was increased proportionally with the increase of influent concentration. In primary sedimentation tank, organic and inorganic components in suspended solids were coprecipitate when SS was removed, and excessive removal of organic matter occurred during the removal of suspended inorganic matter. In the case of high concentration of SS, the synergistic efficiency for the removal of COD and ISS was more obvious. Therefore, the wastewater treatment plant showed higher removal efficiencies of COD, SS, and ISS.

The value of SS/COD for the influent in the grit chamber of the wastewater treatment plant was about 1.78, which was converted to BOD_5_/COD was 0.45 according to the typical domestic sewage to [11], and the value of SS/BOD_5_ for the influent was 3.96. Compared with the value of SS/COD (1.1) in developed countries, the value of SS/COD for the influent in the wastewater treatment plant was high. After the primary sedimentation treatment, the value of SS/COD was reduced to 1.14, which was converted to SS/BOD_5_ was 2.53 and still higher than 1.1. After primary sedimentation treatment, the value of ISS/COD for influent was reduced from 1.3 to 0.93, which was still much higher than the value of 0.2 in developed countries. The results indicated that a large amount of inorganic solids entered the biological treatment structure, which might be the reason for the decrease of MLVSS/MLSS in the wastewater treatment plant. After treatment of primary sedimentation tank, the value of COD/TN was decreased from 9.3 to 6.11, becoming a typical low-carbon source wastewater [12–14]. At present, in order to solve the problems of carbon source required for phosphorus and nitrogen removal in most wastewater treatment plants, the primary sedimentation tank had been generally eliminated in small and medium-sized urban sewage plants using SBR and oxidation ditch. According to the research results, it was suggested that the primary sedimentation tank should be retained in wastewater treatment plants with high concentration of inorganic suspended solids in influent, and the carbon source was retained by hydrolysis and fermentation of wastewater in the primary sedimentation tank.

### 3.2. Analysis of Low Removal Efficiency of Inorganic Solids in Wastewater Treatment Plant

According to the above results, the primary sedimentation tank showed high removal efficiencies for ISS and SS and up to 69.71% and 69.86%, respectively, but the removal efficiencies for SS and ISS were only 6.68% and 4.91%, respectively. Therefore, the main reason for the low removal efficiency of inorganic solids in the pretreatment system was the lower removal capacity of sand in the sedimentation tank. Generally, the sediment was designed to remove silt with a relative density of 2.65 and particle size larger than 0.2 mm, but the removal performance of silt with particle size less than 0.2 mm was not good [15]. The removal efficiency of a typical grit chamber on sand with different particle sizes under optimal operating parameters is shown in Table 3.

The above results about removal efficiency of grit were achieved basing on the optimal operating parameters and skilled operation by the American Water & Wastewater Institute. There was a great difference about the operation effect of rotational flow grit chamber between foreign report and research in our country, and it was difficult to achieve the higher removal efficiency of sand in domestic grit chamber [16, 17].

The combined drainage system was adopted in the area that the wastewater treatment plant belonging to; meanwhile, the service area was large, and the sewage pipe network was long. Therefore, inorganic particles with large particle size were easy to deposit in the sewage pipe, resulting in small particle size of inorganic particles entering the wastewater treatment plant [18, 19]. The average particle size was only about 60 *μ*m, which was much lower than 100 *μ*m, so the removal efficiency of sand under the optimal operating parameters was less than 75%. However, the removal efficiency of the sand in grit chambers was lower than 7% and far below than the design level coupled with the gap between the actual control level of the wastewater treatment plant and the operation process, resulting in the lower removal efficiency of the sand in grit chambers for the wastewater treatment plant.

Rotational flow grit chamber was used in this wastewater treatment plant and the blade speed needed to adjust in order to achieve the high removal efficiency of grit [20]. In addition, the head loss in the tank was a function of the size of sediment to be removed. So the head loss should be increased accordingly in order to remove smaller particles, but there was no clear and feasible operation method for the adjustment of speed and water level. The HRT of rotational flow grit was short, and the flow rate had strict requirements, so it was greatly affected by water fluctuation. Therefore, it was the key to improve the capacity of wastewater treatment plant to deal with the inorganic solids through diversion of rainwater and sewage and strengthen the operation control of grit chamber.

### 3.3. Annual Variation of MLVSS/MLSS

The annual variation of MLVSS/MLSS is shown in Figure 2. MLVSS/MLSS ranged from 0.4 to 0.6 from January to March, reached the maximum value of 0.57 in February, and then gradually decreased to the lowest value of 0.24 at the end of September.

According to outdoor drainage design specifications (GB50014-2006), the sludge concentration of A^2^/O process should be controlled between 2500 and 4500 mg/L when the MLVSS/MLSS of the mixture could be stabilized at the normal level (about 0.7), that was, the MLVSS concentration should be controlled between 1750 and 3150 mg/L [13]. The sewage plant must obtain a higher concentration of sludge to maintain the MLVSS at the normal level when MLVSS/MLSS was much lower than 0.7. During the rainy season, the sludge in this sewage plant showed a high concentration of inorganic substances and it must be maintained at a high sludge concentration. The value of MLVSS/MLSS was increased from January to March, so the sludge concentration was appropriately reduced. Meanwhile, the average concentration of sludge was about 4811 mg/L, and MLVSS/MLSS was about 0.49, so the concentration of MLVSS was about 2357 mg/L. Similarly, the concentration of MLVSS in rainy season was 1900 mg/L. After increasing the concentration of sludge, the concentration of organic matter for sludge in the sewage plant meets the requirements of “Code for design of outdoor drainage.” Although the sewage plant can maintain the normal operation of the sewage treatment system by increasing the concentration of sludge, the inorganic solids in the influent might be accumulated in the sewage treatment system. The inorganic solid suspended in the mixture increased the density of sludge, which led to the difficulty of mechanical mixing or aeration, blockage of sludge pipes, aggravation of mechanical wear of pipes, and dehydration equipment. Therefore, it would increase energy consumption and operating costs [14, 21, 22].

## 4. Conclusions

High concentration of inorganic suspended solid and low treatment efficiency of inorganic suspended solid for the pretreatment system were the common problems in wastewater treatment plant. The low removal efficiency of ISS was ascribed to the weak removal efficiency of sand in the sedimentation tank after long tome analysis, while the primary sedimentation tank showed a higher removal efficiency of sand. Therefore, it was suggested that the wastewater treatment plant with high concentration of inorganic suspended solids in influent should retain the primary sedimentation tank and strengthen the operation regulation of the grit chamber.

## Figures and Tables

**Figure 1:** Sampling points of the wastewater treatment plant.

**Figure 2:** Annual variation of MLVSS/MLSS.

**Table 1:** Average concentration of pollutants at each sampling point.

Index	Influent of grit chamber	Influent of primary sedimentation tank	Effluent of primary sedimentation tank
Particle size (*μ*m)	60.93 ± 7.17	57.58 ± 8.15	49.56 ± 7.73
COD (mg/L)	635 ± 203	620 ± 177	277 ± 91
SS (mg/L)	1123.2 ± 272.7	1048.7 ± 335.7	317.6 ± 125.0
ISS (mg/L)	809.2 ± 234.5	769.5 ± 261.3	231.9 ± 86.9
TN (mg/L)	67.72 ± 8.23	64.24 ± 9.13	45.08 ± 8.22
TP (mg/L)	9.3 ± 1.4	8.7 ± 1.4	4.8 ± 1.1
ISS/COD	1.34 ± 0.40	1.30 ± 0.51	0.93 ± 0.89
COD/TN	9.30 ± 2.29	9.61 ± 2.24	6.11 ± 1.59

**Table 2:** Removal efficiency of pretreatment system.

Structures	Removal efficiency of pollutant (%)				
	COD	SS	ISS	TN	TP
Grit chamber	2.36	6.68	4.91	5.14	6.45
Primary sedimentation tank	55.32	69.71	69.86	29.82	44.83

**Table 3:** The removal efficiency of grit with different particle size by two kinds of grit chambers.

Particle size (*μ*m)	350	250	200	150	100
Removal efficiency of grit using rotational flow grit chamber (%)	95	92	90	85	75
Removal efficiency of grit using aerated grit chamber (%)	92	80	95	42	0

## Data Availability

The labeled dataset used to support the findings of this study is available from the corresponding author upon request.
